The article "SWOT Approach for Audience Online Conversion Rate: An Applied Research on Scenic Spot Projects" was published in 2022. Journal: J Environ Public Health.

# SWOT Approach for Audience Online Conversion Rate: An Applied Research on Scenic Spot Projects

**DOI:** 10.1155/2022/7795524

**Published:** 2022-07-18

**Authors:** Jiaran Ding

**Affiliations:** ^1^Chengdu Jincheng College, Chengdu 611731, China; ^2^Jiangxi University of Technology, Nanchang 330098, China; ^3^SEGi University, Kuala Lumpur 47810, Malaysia

## Abstract

With the rapid development of social economy and people's increasing requirements for spiritual life, tourism projects are booming. At the same time, in order to improve their competitiveness, tourism regions also pay great attention to the attraction of performing arts projects to the audience, especially the online conversion rate. The original online conversion rate survey method cannot effectively judge the online conversion, and the comprehensive judgment ability is weak. At present, there is a lack of necessary analysis methods in the research of audience online conversion rate, so the research results cannot meet the actual requirements. Moreover, there are some deficiencies in the research depth of conversion rate at home and abroad. In order to shorten the abovementioned gap, comprehensive analysis methods should be applied to focus on online transformation. Based on the abovementioned reasons, this paper proposes a method based on SWOT to build a prediction model of audience online conversion rate. First, SWOT is used to cluster the data of strengths, weaknesses, potential dangers, and competitors and sort the data to judge the importance of different data, so as to improve the accuracy of the online conversion rate judgment results of viewers. Then, SWOT classifies the data to form analysis particles in different aspects and analyzes the co-evolution and optimal results of analysis particles in different aspects. After a simulation test, the SWOT model constructed in this paper is superior to the online conversion rate survey method in terms of calculation accuracy and calculation time and the overall effect is higher. At the same time, the integration of threshold, weight, and other adjustment functions further enhances the analysis effect of SWOT model. Therefore, a SWOT model can accurately and quickly predict the online conversion rate of audience.

## 1. Introduction

At present, the state has put forward the concepts of online reservation and online marketing, and major tourism institutions and local governments attach great importance to the evaluation of online conversion rate. In order to meet the national policies and calls, various places have carried out the analysis of audience online conversion rate. The analysis of audience online conversion rate can not only judge more accurately, so as to obtain accurate data, so as to arrange scenic spots, but also save a lot of human resources. Therefore, in-depth analysis of audience online conversion rate has the dual significance of saving scenic spot cost and corresponding national call. Moreover, studying the online conversion rate of audience can improve the popularity and comprehensive potential of scenic spots. According to the survey data of tourism performance development in 2022 Zhao M. L. [1], the online conversion rate of visitors is increasing year by year, as shown in Figure 1.

In this case, the demand for audience online conversion rate analysis is increasing, and permeates all aspects of entertainment and performing arts projects. Domestic tourism research institutions pay great attention to the problem of audience online conversion rate and make corresponding data statistics Zakeri S. [2]. At present, the SWOT method is mainly used in the commercial field, but there are few research studies in the performing arts field and online field, and there is a lack of corresponding practical cases. The problem of the audience online conversion rate is a comprehensive research problem, which focuses on the actual investigation and analysis. At present, the online conversion rate of audience is too quantitative, and there are few comprehensive research results. The SWOT method can be a more comprehensive analysis, not only quantitative analysis, but also qualitative research. Therefore, it is technically feasible and theoretically feasible to use the SWOT method for analysis; the SWOT analysis of audience online conversion rate is a comprehensive analysis, which can not only predict audience's psychology but also analyze and judge according to behavior, so the analysis of audience online conversion rate is more comprehensive. SWOT has its own advantages. It can obtain the data needed for analysis through a large number of data surveys and actual case studies. However, SWOT also has some disadvantages, that is, it is difficult to obtain data, and a large number of data should be collected in the early stage. Foreign scholars have applied the SWOT theory to online analysis, art, and other fields and achieved good results, but the above analysis results do not meet the domestic requirements, so it is necessary to comprehensively analyze the audience online conversion rate according to SWOT. Therefore, on the basis of previous research, this paper constructs a SWOT prediction model of audience online conversion rate, which not only provides support for the accurate analysis of audience online conversion rate but also enriches relevant theories.

Because the online conversion rate of audience involves threats, potentials, competitions, advantages and other aspects and presents a nonlinear relationship; the SWOT model is constructed to analyze the relevant data in a semistructured way, which accurately reflects the mapping characteristics among various factors. In SWOT analysis, through repeated iterative analysis by Wang Y. [3], the data of audience online conversion rate can be better processed, and the nonlinear analysis requirements can be realized. Some domestic scholars have built a prediction model of SWOT audience online conversion rate by Shimizu K. [4] to analyze the audience online conversion rate. The results show that SWOT has a high analysis effect on each index of audience conversion rate Saxena V. [5].

SWOT is a qualitative analysis method, which integrates the learning mechanism of quantitative analysis to make fuzzy analysis of online transformation problems. First, based on SWOT, we initialize the online conversion rate of the audience Savari M. [6] and simplify the content of the data. In previous studies, (1) mainly adjust the four parameters of SWOT, and then compare it with the online conversion rate index of audience, so as to realize single index and multi index analysis in a certain stage Qasim Q. I. [7]; (2) build the audience online conversion rate set and classify the data in the set Pandyaswargo A. H. [8]. Finally, time division is carried out according to the weight of classification to improve the accuracy of SWOT analysis Panayotova M. [9]; and (3) compare with other intelligent analysis models, such as the Bayesian theory and grey theory, to verify the accuracy of the model Nair A. S. [10].

## 2. Related Concepts

### 2.1. SWOT Theory

SWOT is a qualitative analysis method, which mainly solves four problems: threat, strength, weakness, and potential Miura, S. I. [11], and is widely used in management, industry, art and other fields. SWOT includes strengths, weaknesses, potential competition, and threats. SWOT is a quantitative analysis method, which can investigate and inspect the research content and obtain necessary data resources. At the same time, SWOT can comprehensively analyze the data resources under investigation through subjective judgment, and analyze them more comprehensively and carefully, so as to improve the accuracy of analysis results. Simply put, SWOT can not only avoid the errors of subjective analysis but also improve the accuracy of quantitative analysis, so SWOT is widely used in various fields, especially in the field of online analysis. SWOT is superior in nature and describes qualitative data continuously Miller, E. [12]. At the same time, irregular points are randomly selected for cyclic analysis to improve the accuracy of calculation results Meza, A. [13]. If *H*_*it*_ represents the online transformation set of *i* viewer *t* time, and *x* belongs to *H*_*ij*_.

Suppose 1: *Z*_*j*_(*x*)=∪∑_*i*,*t*=1_^*n*^{*x*_*it*_^*j*^*·ω*⇄*φ*(*k*)}, *ω* ∈ (1, ⋯*n*), Δ*φ*(*k*)=∑Δ*C*(*x*, *ε*), then *Z*_*i*_(*x*) is the best online transformation set. Where, Δ*C*(*x*, *ε*) is the adjustment coefficient *ε* of the number of viewers *x* and the conversion result. Among them, *ε* is the key point of SWOT analysis. When *x*_*it*_=∮(tan  2/∑sin(*πt*/*ρ*)), and *ρ* is the minimum prime number of online conversion. If 2*s*∑sin(*πt*/*ρ*) < ∑_*i*,*j*,*t*=1_^*n*^*ω*{*x*_*j*_^*it*^*·k*, the online conversion list in SWOT is the best, as shown in Figure 2.

The relevant theories of SWOT are as follows:

**Theorem 1 .**

*Z*_*n*_(*x*) is the potential hazard, and *φ*(*x* · *k*) (note: it is the potential hazard judgment function of *t* time), then the calculation formula of the conversion rate judgment function is as shown in Formula (1).

(1) $$\begin{array}{c} \int_{x\in G_{ij}}f\left(x\right)dx-\bar{\overset{n}{\underset{j=1}{\sum }}f\left(P_{j}\left(x\right)\right)}<Q\left(f\left(x\right)\right)\cdot \varphi \left(k\right). \end{array}$$

Among them, the global conversion rate is judged for.

**Theorem 2 .**

If the following conditions *f*(*x*) are satisfied, *f*(*x*) < *ε*, *f*(*x*)′ < *ε*,… *f*(*x*)^*j*^ < *ε*, then any function value on the right side of the time series is within the integral *f*(*x*), and the error of judging data by the right conversion rate is less than lin(1/*x*).

**Theorem 3 .**

Assuming that any audience is randomly distributed in various regions, the calculation formula of the deviation between tourism performance (*δy*/*δx*)(*x*) and audience demand is as follows (2).

(2) $$\begin{array}{c} \frac{\delta y}{\delta x}\left(x\right)=\prod \underset{\delta x⟶0}{\lim}\left(\sqrt{\left(Z_{ij}\left(x\right)\right)}.\right) \end{array}$$

Among them, (*δy*/*δx*)(*x*) is between collections [0, +*∞*].

From Theorems 1 and 2, it can be seen that the derivative of SWOT can convert the error change of the judgment result, which has nothing to do with the audience *i* and the time *t*. Therefore, the SWOT model provides a good theoretical basis for multifaceted analysis, and the influence of subjective changes of audience on judgment results Mello, J. [14].

According to Theorem 3, the local deviation of the data in SWOT is , lim_*δx*⟶0_(Δ*s*) the average value of the deviation is $\prod \lim_{\delta x⟶0}\left(\sqrt{\left(Z_{ij}\left(x\right)\right)}\right)/\sum Z_{ij}\left(x\right)$, which indicates that the local deviation is less than the uniformly distributed deviation, and the SWOT model can judge the amplitude constraint of the right conversion rate. Combining SWOT with the fuzzy algorithm, this paper puts forward the control of the judgment range of conversion rate, and the more it is, the better the ability of SWOT to correct the wrong data. At the same time, this paper makes a multidimensional analysis of the audience online conversion rate, forms an initial particle swarm, and makes a continuous analysis of the audience online conversion rate. The result is shown in Figure 3.

### 2.2. SWOT's Analysis of Audience Online Transformation

SWOT is a clustering method, which can make the audience online transformation fuzzy and adaptive, and make up for the lack of audience online transformation data Long, Y. [15]. SWOT realizes comprehensive analysis by constantly revising the set and making “if” judgment. The conditions of SWOT analysis are shown in Table 1 below:

Among them, *λ*(*x*_*i*_) is a satisfaction analysis function, *g*_*ij*_ is transformation set, *M*(*x*) is constraint function Li K. [16], ∏*M*(*x*_*i*_) · *λ*(*x*_*i*_) is relationship between satisfaction and transformation, and *y* is transformation evaluation result. The input data of SWOT model are unstructured data, part of which is missing and part of which is complete, so it can be judged and analyzed by the rough set method Lawinska O. [17].

Assuming that any viewer is, *x*_*i*_ under the constraint rule *M*, the relationship *x*_*i*_ with *y*_*i*_ the transformation result can be obtained, as shown in formula (3).

(3) $$\begin{array}{c} C\cdot g_{ij}=\sum_{i,j=1}^{n}\underset{\delta x⟶0}{\lim}x\forall c|\frac{\left(x_{i}⇄c_{ij}\right)}{b_{ij}}. \end{array}$$

Among them, *x*_*ij*_ and *b*_*ij*_ are, respectively, the audience and expectation of online transformation of audience; *C* is the adjustment coefficient of transformation Islam A. [18], and set *g*_*ij*_ is the data set of performance items.

According to formula (3), integration *δ* is the adjustment coefficient of transformation, and *k* is the uncertainty factor in the transformation process. According to the calculation method of online conversion rate, the online conversion result can be obtained, as shown in formula (4).

(4) $$\begin{array}{c} y=∡\frac{\sum_{ij}^{k}g^{k}\left(x\right)⇄f\left(P_{j}\left(x\right)\right.}{\text{mean}\sum_{i,j=1}^{n}g_{ij}^{k}\left(x\right)}|k. \end{array}$$

The SWOT model shortens the processing time of online conversion rate, reduces the initial data processing amount, and improves the data processing speed by analyzing indicators such as threat and potential Hosseinnejad A. [19]. At the same time, SWOT reduces the influence of external interference on the results and realizes the “reasonable switching” of different audiences, so that the results are more in line with the actual requirements Hosseini S. M. [20].

## 3. SWOT Model Construction

### 3.1. Initialization of Relevant Parameters

The SWOT model takes into account the advantages of multidimension and overall situation, which can improve the analysis ability of qualitative data and comprehensively carry out online conversion rate analysis. The SWOT model realizes evolutionary analysis of initial sequence and multidimensional sequence and uses threshold and weight factor to realize iterative analysis between audience and online conversion, and finally obtains the optimal value of conversion rate judgment.

### 3.2. Initialization of SWOT

SWOT analysis of money, all data should be in a random distribution. If the ranking uncertainty is strong, that is, nonnormal distribution Grillini V. [21], which belongs to discrete distribution; there will be local “traps”, which will reduce the calculation accuracy of the global optimal solution and increase the error rate of the calculation results. In order to enhance the normality of the sequence Gago D. [22], it is necessary to expand the scale of the sequence and expand the scope of audience analysis of performing arts projects. The results are shown in Figure 4.

Figure 4 shows the random distribution structure of SWOT data, and the number of visitors reaches 50. Through comparison, it is found that the data of threats, opportunities, and advantages have a strong random distribution, which meets the requirements of calculation. In addition, the online transformation model constructed by SWOT has nothing to do with the geographical location of the audience and is suitable for data processing in different ranges. Moreover, when taking points each time, the distribution effect of the initial data is the same, and the stability of the data set is high. It is consistent with the audience distribution of the actual performance project.

### 3.3. Collaborative Processing of Multiple Strategies

SWOT needs a comprehensive judgment, and it is also an important measure to measure the online transformation of viewers. In the initial stage of SWOT calculation, we should not only pay attention to global search but also carry out collaborative analysis of different indicators. In order to improve the SWOT computation efficiency of the algorithm, this paper needs multistrategy cooperation, so that the strengths, weaknesses, and threats can be repeatedly calculated; finally, accurate results can be obtained Boitrelle F. [23].

(1) Group behavior pattern, the calculation is as shown in formula (5).
  (5) $$\begin{array}{c} y_{ij}\left(t+1\right)=\frac{\left[\delta \cdot \sum_{i,j,k=1}^{n}g_{ij}^{k}\left\{x\left(t\right)⇄f\left(P_{j}\left[x\left(t\right)\right]\right.\right\}\right.}{\prod g_{ij}^{k}\left[x\left(t\right)\right]}. \end{array}$$
(2) Advantage and disadvantage judgment mode, the calculation is as shown in formula (6).
  (6) $$\begin{array}{c} y_{ij}\left(t+1\right)=\left|\frac{\left[\delta \cdot \sum_{i,j,k=1}^{n}g_{ij}^{k}\left\{x\left(t\right)\cdot f\left(P_{j}\left[x\left(t\right)\right]\right.\right\}\right.}{\max\prod g_{ij}^{k}\left[x\left(t\right)\right]}⇄\frac{\left[\delta \right.\cdot \sum_{i,j,k=1}^{n}g_{ij}^{k}\left\{x\left(t\right)\cdot f\left(P_{j}\left[x\left(t\right)\right]\right.\right\}}{\min\prod g_{ij}^{k}\left[x\left(t\right)\right]}\right|. \end{array}$$
(3) Fusion mode, the calculation is as shown in formula (7).
  (7) $$\begin{array}{c} y_{ij}\left(t+1\right)=\frac{\left[\delta \cdot \sum_{i,j,k=1}^{n}g_{ij}^{k}\left\{x\left(t\right)⇄f\left(P_{j}\left[x\left(t\right)\right]\right.\right\}\right.}{\max\prod g_{ij}^{k}\left[x\left(t\right)\right]}. \end{array}$$

Among them, *c*_*i*_ is synergy coefficient, *r*_*i*_ is correlation coefficient, *ω* is average weight and *n* is transformation strategy.

In this paper, the SWOT model is improved in two aspects. On the one hand, it expands the search range of online audience. After each iterative calculation, the factors in SWOT will be calculated repeatedly. At the same time, it keeps the diversity of different audiences and increases the possibility of local calculation. On the other hand, the convergence of strengths and weaknesses improves. In order to improve the global search ability of SWOT, nonlinear adjustment coefficient and linear weight are integrated, and the specific calculation formula is as formula (8).

(8) $$\begin{array}{c} \alpha =\forall t,T|\frac{{\text{Line}}_{t}^{d}\cup 1}{{\text{Line}}_{T}^{D}}, \end{array}$$

where *E* is the constraint coefficient, *T* is the calculation time, *T* is the maximum calculation time, and *D* is the iteration times. In the initial stage of SWOT, there are many constraints, which can improve the accuracy of global calculation. In the middle and later period of calculation, there are fewer constraints, which can shorten the calculation time of local optimal value. The specific calculation is as shown in the following formula.

(9) $$\begin{array}{c} \xi ={\sum_{d=1}^{D}\left[\frac{\left(w_{\max}\cup \sum_{t=1}^{T}\Delta w_{i}\right)}{\left(\sum_{t=1}^{T}\Delta w_{i}\subseteq w_{\min}\right)}\right]}^{d}. \end{array}$$

Among them, *w*_max_ and *w*_min_ are the maximum and minimum weights respectively, which mainly limit the search scope.

### 3.4. Judgment Process of Audience Online Conversion Rate Based on SWOT

The basic idea based on SWOT is a multiangle comprehensive analysis. First, we set the initial value and threshold [17], and then calculate the optimal solution to improve the calculation accuracy of the optimal solution. The results are shown in Figure 5.

**Step 1 .**

Identify the needs to focus on online transformation problems and determine the relevant data structures. Initialize the whole data set and set weights and thresholds. According to SWOT, we determine the iteration times of this paper;

**Step 2 .**

After the data are initialized, set the parameters. The maximum analysis audience *n* = 100, the maximum weight = 0.6, the minimum weight *w*_min_=0.4, and the synergy constant max between different aspects max *c*_*i*_*c*_2_=3.32.

**Step 3 .**

Generate the moderation function. Using the SWOT theory, the coordination coefficient of SWOT is adjusted constantly, and the accuracy of each SWOT is obtained to obtain a moderate function.

**Step 4 .**

Search the optimal position of SWOT and the optimal position of each subgenetic particle globally.

**Step 5 .**

Iteration of optimal position and speed. In the SWOT model, nonlinear adjustment coefficient *α* and linear weight are *ω* added.

**Step 6 .**

All subsequences co-evolve at the same time. After one iterative calculation is completed, the optimal global calculation position is selected and shared with other subsequences. Other subsequences iterate gradually to this position, so as to get the best position result.

**Step 7 .**

Judge whether the maximum iteration number is reached, and return the results of threshold, weight, optimal position, etc.

## 4. Practical Case Analysis

### 4.1. Performance Judgment of SWOT Model

To verify the performance of the SWOT model, the following analysis is performed. Because there are many data types of audience online conversion rate, in order to make a better comprehensive analysis, it is necessary to transform the corresponding data. Unstructured data are standardized by classification, and structured data are processed by enlarging and reducing actual data, so as to obtain the same analysis data. The sphere is the globally unique minimum function [18], as follows:

(10) $$\begin{array}{c} F_{1}\left(x\right)=\min\sum_{i=1}^{n}\left[x_{i}^{2}\right]. \end{array}$$

RastrinH Cosine Modulation Transfer Function verifies the practicability of the model solution [19]; the formula is as follows:

(11) $$\begin{array}{c} F_{2}\left(\left(x\right)\right)=\prod x_{i}^{2}⇄10\;\cos\left(2\pi x_{i}\right). \end{array}$$

Ackley is a multidimensional point function that tests the speed at which multidimensional data is computed, which is formulated as follows:

(12) $$\begin{array}{c} F_{3}\left(x\right)=\text{lin}\left\{-0.2\oint \sqrt{\frac{1}{n}\sum_{i=1}^{n}x_{i}^{2}}\right\}⇄\;\exp\;{\left\{\frac{1}{n}\sum_{i=1}^{n}\cos\left(2\pi x_{i}\right)\right\}}^{20}, \end{array}$$

where *N* is the total number of indicators for calculating data, *x*_*i*_ is any audience. *x*_*i*_ value range {−100, 100}. In order to facilitate the calculation, the number of spectators in SWOT in this paper is *n* = 100, and the longest data collection time is *t* = 12 months. The above three function tests are carried out and the average results are taken. The specific calculation results are shown in Table 2.

The convergence diagram of each data in Table 2 is shown in Figures 6–8.

It can be seen from Table 1 that compared with the investigation method, the SWOT and statistical method algorithms proposed in this paper are closer to the global optimal value. In terms of standard deviation, average value, and value range, the SWOT algorithm is better than the other two algorithms. According to the curve changes in Figures 6–8, the SWOT algorithm has a better stability and faster convergence speed. Therefore, the SWOT algorithm has better convergence speed, calculation accuracy, and summation stability. The calculation results are shown in Table 3.

### 4.2. Case Data and Preprocessing

The sample data of this paper select the online conversion rate samples of 2021 viewers in tourism performing arts companies from December 12, 2019 to March 4, 2021. Among them, from March 4, 2019 to January 12, 2020, some data were missing due to human operation, and the default value was used to make up for it in the later period [21].

The prediction data set of audience online conversion rate includes digital behavior, bionic behavior, natural behavior, psychological behavior, and expected behavior [22]. After preliminary data preprocessing, 1982 lines of structured data and 38 lines of semistructured data are obtained. In order to facilitate data analysis, the online conversion rate of audience is divided into five levels: complete conversion, basic conversion, general conversion, no conversion, and no conversion at all. The processing results of data volume are shown in Table 4.

Due to the lack of some data in this paper, the data from December 12, 2019 to January 24, 2021 are taken as the training set, with a total of 421 pieces; the data from January 25, 2021 to March 4, 2021 are used as test sets, with a total of 102 pieces. The training results of each data are shown in Figure 9.

### 4.3. Test Results

To verify the SWOT algorithm proposed in this paper, we compare the results with the statistical method and the investigation method, and the results are shown in Figure 10.

It can be seen from Figure 7 that the accuracy of the SWOT algorithm is higher than the investigation method and statistical method, but the error rate is lower, which shows that the calculation of SWOT, investigation method, and statistical method is relatively stable, while the calculation of SWOT, investigation method and statistical method is uneven. The average results of the above three algorithms are shown in Table 5.

It can be seen from Table 5 that the qualitative online conversion rate survey method has the problems of insufficient accuracy and large variation of calculation results in different levels. Compared with the qualitative online conversion rate survey method, the accuracy of SWOT algorithm is significantly improved. At the same time, the accuracy of the SWOT algorithm is greater than 80%, which is better than the investigation method. In order to further verify the superiority of SWOT algorithm, the calculation time of different algorithms is compared, and the results are shown in Figure 11.

It can be seen from Figure 11 that the calculation time of SWOT algorithm is shorter, and the optimization result is more significant Baez-Leon, C. [24]. The reason is that SWOT increases the synergy coefficient, weight and convergence factor in threats, strengths, and weaknesses, which can make a more comprehensive analysis of the audience online conversion rate.

## 5. Concluding Remarks

In this paper, the SWOT theory is proposed, and combined with a multidimensional coevolution method, the online conversion rate is analyzed from the aspects of advantages S. Amirshenava, and M. Osanloo [25], disadvantages, and potential. In order to make the analysis results more accurate, we set the threshold and weight and build a SWOT analysis model A. Islam W. A. Al-Kutti M. Nasir Z. A. Kazmi and M. Sodangi [18]. The results show that compared with the investigation method, statistical method, and SWOT online conversion rate investigation method, its prediction accuracy and calculation time are better, and it can accurately judge the online conversion rate of the audience. However, in the SWOT model, there is a lack of dynamic analysis of potential advantages and threats A. Meza M. Koc and M. S. Al-Sada [13], resulting in a certain timeliness of the results and unable to make long-term prediction. Therefore, in the future research, the dynamic function will be integrated to prolong the prediction time of audience online conversion rate.

## Figures and Tables

**Figure 1:** Audience online conversion rate of tourism performance projects.

**Figure 2:** Results of SWOT online transformation.

**Figure 3:** Continuity analysis of the online conversion rate.

**Figure 4:** Initial SWOT sequence constructed by the random method.

**Figure 5:** Calculation flow chart based on SWOT.

**Figure 6:** Convergence result of Sphere function optimization.

**Figure 7:** Convergence result of RastrinH function optimization.

**Figure 8:** Convergence result of Ackley function optimization.

**Figure 9:** Data training results from December 12, 2019 to January 24, 2021.

**Figure 10:** Test results of different algorithms.

**Figure 11:** The calculation time comparison of the SWOT and statistical methods.

**Table 1:** Constraints for SWOT.

Judgement	Constraint condition	Constrained content
Advantage	If: *x*_*i*_∀ *g*_*ij*_	*y*=∑_*i*=1_^*n*^*y*_*i*_=∑_*i*=1_^*n*^*M*(*x*_*i*_) · *λ*(*x*_*i*_)
Weak	If: *x*_*i*_∩*g*_*ij*_	*y*=∏*M*(*x*_*i*_) · *λ*(*x*_*i*_)
Threat	If: *x*_*i*_ ∪ *g*_*ij*_	*y*=lim_*δx*⟶0_*M*(*x*_*i*_) · *λ*(*x*_*i*_)
Opportunity	If: *x*_*i*_⇄*g*_*ij*_	*y*=(*δy*/*δx*)*M*(*x*_*i*_) · *λ*(*x*_*i*_)

**Table 2:** Test results of different test functions.

Detection function	Algorithm	Value range	Average difference	Standard deviation	Global optimal solution
Sphere	SWOT	ln 1.99	ln 5.96	ln 2.98	1
	Investigation method	ln 4.96	ln 1.99	ln 2.98	
	Statistical method	ln 3.97	ln 1.99	ln 5.96	

RastrinH	SWOT	ln 3.97	ln 2.98	ln 1.99	1
	Investigation method	ln 5.96	ln 5.96	ln 3.97	
	Statistical method	ln 3.97	ln 4.96	ln 3.97	

Ackley	SWOT	ln 5.96	ln 3.97	ln 5.96	1
	Investigation method	ln 1.99	ln 4.96	ln 3.97	
	Statistical method	ln 4.96	ln 4.96	ln 1.99	

**Table 3:** Test results of different algorithms.

Algorithm	Average	Standard deviation	Value range
SWOT	(34.41, 38.71, 33.33)	(37.5, 41.67, 39.58)	(3.33∼7.5)
Statistical method	(37.63, 35.48, 38.71)	(39.58, 40.63, 31.25)	(3.33∼6.46)
Investigation method	(41.94, 37.63, 32.26)	(37.5, 31.25, 34.38)	(5.42∼37.5)

**Table 4:** Classification and proportion of audience online conversion rate.

Transformation grade	Amount of data	Proportion (%)
Complete transformation	223	12.38
Basic transformation	843	24.95
General	521	8.81
Cannot convert	42	0.37
Completely unable to transform	172	0.76

**Table 5:** Comparison of prediction accuracy of different grades.

Transformation grade	Complete transformation	Basic transformation	General	Cannot convert	Completely unable to transform
SWOT	(40.86, 36.56, 39.78)	(38.54, 32.29, 40.63)	(6.46, 5.42, 2.29)	(40.86, 36.56, 39.78)	(36.56, 43.01, 38.71)
Investigation method	(40.86, 34.41, 39.78)	(40.63, 33.33, 35.42)	(1.25, 5.42, 0.63)	(40.86, 34.41, 39.78)	(33.33, 39.78, 36.56)
Statistical method	(41.94, 43.01, 41.94)	(31.25, 34.38, 36.46)	(1.67, 8.54, 6.46)	(41.94, 43.01, 41.94)	(36.56, 38.71, 32.26)

## Data Availability

The data used to support the findings of this study are available from the corresponding author upon request.

## References

[1] Zhao M. L., Zhou J., Kan U., Mu J. (2021). SWOT research on the development of rural tourism E-commerce system under the background of big data era. *Mobile Information Systems*.

[2] Zakeri S., Konstantas D., Sink Z., Cheikhrouhou N. (2022). The grey ten-element analysis method: a novel strategic analysis tool. *Mathematics*.

[3] Wang Y. (2022). Research on the development mode of ecotourism in XI’an based on the SWOT analysis model. *Fresenius Environmental Bulletin*.

[4] Shimizu K. (2021). A SWOT analysis of the guidelines on prevention of HIV/AIDS in Japan in the context of COVID-19. *Infectious Disease Reports*.

[5] Saxena V., Bahurupi Y., Mishra M., Singh A., Parate S., Sandhu H. (2022). Strength, weakness, opportunities, and threats (SWOT) analysis of virtual outpatient department under telemedicine department during the COVID-19 pandemic. *Cureus*.

[6] Savari M., Amghani M. S. (2022). SWOT-FAHP-TOWS analysis for adaptation strategies development among small-scale farmers in drought conditions. *International Journal of Disaster Risk Reduction*.

[7] Qasim Q. I. (2021). The influence of the SWOT analysis strategy on the achievement of the fifth preparatory literary class students’ evaluative thinking at history. *International Journal of Early Childhood Special Education*.

[8] Pandyaswargo A. H., Wibowo A. D., Maghfiroh M. F. N., Rezqita A., Onoda H. (2021). The emerging electric vehicle and battery industry in Indonesia: actions around the nickel ore export ban and a SWOT analysis. *Batteries*.

[9] Panayotova M., Krastanov J., Varlyakov I., Stoyanchev T., Marinov I. (2021). SWOT analysis for supporting development of the grazing livestock meat production sector in Bulgaria through the GREENANIMO project activities. *Bulgarian Journal of Agricultural Science*.

[10] Nair A. S., Kumar N., Indu J., Vivek B. (2021). Monitoring lake levels from space: preliminary analysis with SWOT. *Frontiers in Water*.

[11] Miura S. I., Nose D., Kanamori K., Imaizumi S., Shimura H., Saku K. (2021). Sustainable hospital management by a cross SWOT analysis in a medium-sized hospital. *Sustainability*.

[12] Miller E., Reddy M., Banerjee P. (2022). Strengthening institutions for public health education: results of an SWOT analysis from India to inform global best practices. *Human Resources for Health*.

[13] Meza A., Koç M., Al-Sada M. S. (2022). Perspectives and strategies for LNG expansion in Qatar: a SWOT analysis. *Resources Policy*.

[14] Mello J. A. V. B., Pinto B. G. J., Mello A. J. R. (2022). SWOT analysis and GUT matrix for business management and problem solving: an application in a Brazilian case. *Cuadernos De Gestion*.

[15] Long Y., Li Y., Lei X., Hou Y., Guo S., Sun J. (2021). A study on comprehensive evaluation methods for coordinated development of water diversion projects based on advanced SWOT analysis and coupling coordination model. *Sustainability*.

[16] Li K. (2022). SWOT analysis of e-commerce development of rural tourism farmers’ professional cooperatives in the era of big data. *IET Communications*.

[17] Ławińska O., Korombel A., Zajemska M. (2022). Pyrolysis-based municipal solid waste management in Poland-SWOT analysis. *Energies*.

[18] Islam A. B. M. S., Kutti W. A., Nasir M., Kazmi Z. A., Sodangi M. (2022). Potential use of local waste scoria as an aggregate and SWOT analysis for constructing structural lightweight concrete. *Advances in Materials Research-an International Journal*.

[19] Hosseinnejad A., Rassouli M., Jahani S., Elahi N., Molavynejad S. (2021). Requirements for creating a position for community health nursing within the Iranian primary health care system: a SWOT analysis. *Frontiers in Public Health*.

[20] Hosseini S. M., Paydar M. M., Triki C. (2021). Implementing sustainable ecotourism in Lafour region, Iran: applying a clustering method based on SWOT analysis. *Journal of Cleaner Production*.

[21] Grillini V., Verlicchi P., Zanni G. (2022). SWOT-SOR analysis of activated carbon-based technologies and O3/UV process as polishing treatments for hospital effluent. *Water*.

[22] Gago D., Mendes P., Murta P., Cabrita N., Teixeira M. R. (2022). Stakeholders’ perceptions of new digital energy management platform in municipality of loulé, southern Portugal: a SWOT-AHP analysis. *Sustainability*.

[23] Boitrelle F., Shah R., Saleh R. (2021). The sixth edition of the WHO manual for human semen analysis: a critical review and SWOT analysis. *Life*.

[24] Baez‐Leon C., Palacios‐Ceña D., de‐las‐Peñas F., Velarde‐García J. F., Rodríguez‐Martínez M. A., Arribas‐Cobo P. (2022). A qualitative study on a novel peer collaboration care programme during the first COVID‐19 outbreak: a SWOT analysis. *Nursing Open*.

[25] Amirshenava S., Osanloo M. (2022). Strategic planning of post-mining land uses: a semi-quantitative approach based on the SWOT analysis and IE matrix. *Resources Policy*.

